The article "The Impact of Cultural Creative Product Design for Sport Events on the Residents' Fitness" was retracted in 2023. Reasons: signs of a paper mill; suspected computer-generated content; unreliable results or conclusions; concerns about the data.

# The Impact of Cultural Creative Product Design for Sport Events on the Residents' Fitness

**DOI:** 10.1155/2022/3150099

**Published:** 2022-09-08

**Authors:** Mohan Li, Yanping Liu

**Affiliations:** School of Art and Design, Harbin University, Harbin 150086, China

## Abstract

Cultural and creative product design of sports events is an important part of sports industry, which can improve the economic benefits of sports industry. Based on this background, this paper puts forward a regression analysis method to deeply analyze the design of cultural and creative products in sports events, aiming at driving the healthy development of residents and improving their health levels. First of all, 620 residents were randomly divided into a control group and an observation group to compare natural characteristics, historical characteristics, folk crafts, regional culture, and other indicators. Then, find out the factors with significant differences, and carry out regression analysis to provide corresponding measures for the design of cultural and creative products in sports events. The results show that the main influencing factors of creative product design are natural characteristics, historical characteristics, folk crafts, regional culture, and promotion effect, and each index has a significant impact on residents' fitness, and there are significant differences. Therefore, all regions should improve the design level of sports events, bring through the development of residents' fitness industry, and effectively guide residents' fitness.

## 1. Introduction

Heilongjiang province attaches great importance to the development of regional culture and the design of cultural and creative products of sports events and takes it as the guide of residents' fitness to promote the improvement of local residents' fitness levels [1]. However, the design of cultural and creative products of sports events needs correct guidance, so as to play a role in promoting residents' fitness. However, some scholars believe that the cultural creative product design of sports events should integrate various factors [2], such as natural characteristics, historical characteristics, folk crafts, and regional culture, otherwise it is difficult to play its role. Some scholars believe that the design of cultural and creative products of sports events needs certain methods as guidance and integration with local cultural characteristics, so as to give full play to the comprehensive advantages of design [3]. At present, there are some controversies in the research of cultural and creative product design for sports events, and there is also a lack of effective methods for evaluation. Therefore, it is an urgent problem for relevant experts to verify the effectiveness of cultural and creative product design of sports events and its role in improving residents' fitness levels. The specific investigation needs are shown in Figure 1.

According to the survey in Figure 1, the demand for cultural and creative product design of sports events changes by 8%, and the actual demand for residents' fitness guidance changes exponentially [4], with an effective guidance demand changing by 14%. The above data show that the promotion demand for residents' fitness guidance is reasonable, and the demand for cultural and creative product design of sports events fluctuates greatly, which further shows that the cultural and creative product design of sports events cannot meet the guidance demand of residents' fitness, and further research will be carried out in the future [5]. Residents' fitness needs are more in the range of 0∼2000, and more concentrated, with a small distribution in the range of 13500∼14000. Therefore, residents' fitness needs show discrete distribution at both ends, which accords with the characteristics of non-normal distribution [6]. This shows that the residents' demand for fitness is increasingly strong and cannot be effectively met, which is a hot issue in current research [7]. It also further shows that the research in this paper meets the current needs and has very important theoretical and practical feasibility. The design of cultural and creative products of sports events should reflect local culture, natural culture, humanistic culture, and other related issues. The cultural and creative product design of sports events is not a single unit, but a regional resident culture [8]. Good cultural and creative product design of sports events can not only enhance the economic status of the region but also arouse the fitness enthusiasm of local residents and promote the improvement of fitness levels [9]. The cultural and creative product design of sports events plays an important role in the cultural construction of the region, and also has a strong impact on the ideology of local residents [10]. Therefore, strengthening the cultural and creative product design of sports events can improve the local sports cultural level and form a good external environment. Some scholars believe that the cultural innovation product design of sports events is only a single product design, which has nothing to do with the humanistic environment, local cultural characteristics, and residents' cultural awareness [11]. It is also believed that the innovative product design of sports events culture is the internal driving force of local economic and cultural development, so it is necessary to strengthen relevant construction and maintain its own sustainable development [12]. At present, there are still some controversies about the cultural innovation product design of sports events and its impact on residents' fitness. Therefore, increasing the research on innovative product design of sports events culture is not only in line with the current research direction but also in line with the current needs of sports culture construction [13]. In addition, the cultural innovation product design of sports events should integrate various factors, It includes not only natural culture, social culture, and folk culture but also other cultures [14], so as to maximize the research scope and depth of culture, promote the sustainable development of innovative product design of sports events culture [15], and play a guiding role in regional economy and residents' fitness consciousness. Based on the above reasons, under the guidance of sports event cultural creativity theory, this paper analyzes the guiding effect of creative product design on residents' fitness and finds out the factors affecting residents' fitness guidance [16]. This paper mainly elaborates on the following aspects: first of all, the cultural and creative products of sports events are analyzed, and the natural characteristics, historical characteristics, folk crafts, and the meaning of regional culture of sports cultural products are discussed, as well as the influence of the above characteristics on residents' fitness; secondly, the problem of residents' fitness is described mathematically [17], and the natural characteristics, historical characteristics, folk crafts, and regional culture of sports cultural products are quantified [18], which lays the foundation for later analysis and; finally, the simulation analysis method is used to verify the effectiveness of the model proposed in this paper, especially the analysis of sports event culture and the impact on residents' fitness, and the research results of this paper are summarized.

## 2. The Research Method of Residents' Fitness Guidance in Product Design

### 2.1. Investigator's Information

A total of 610 residents were selected and divided into general groups and guiding groups according to the research methods. The general situation of each group is shown in Table 1.

In Table 1, there is no significant difference in residents' age, design degree, and guidance, and they all sign the survey consent form, and the survey can be statistically analyzed with the consent of Heilongjiang provincial tourism bureau. From the data in Table 1, it can be seen that there is no significant difference in age, guidance effect, guidance grade, and related indicators between the guidance group and the normal group, indicating that the data of the two groups can be statistically analyzed in the later period. In addition, the age range, guidance grade range, and other related indicators of the two groups are in line with normal distribution, which shows that the selection of data is reasonable and will not have adverse effects on the later results, further indicating the validity of the data. The specific results are shown in Figure 2.

Inclusion criteria: (1) meet the residents' fitness evaluation criteria in the residents' fitness guide proposed by the Ministry of Education; (2) fill in the information less than 30; (3) residents' exercise ability is normal and there are no other related diseases; (4) residents cooperate with relevant research; and (5) residents' bad reputation; exclusion criteria: (1) there are family hereditary diseases; (2) residents have fractures and muscle strains; (3) those with motor disorders; and (4) those, who quit halfway.

### 2.2. Research Methodology

**Assumption 1 .**

The data set is set, the proportion of regional elements in the design of cultural and creative products for each sports event is *f*, the degree of creativity is *t*, the guiding process is *K*, and the product integration factor is *x*_*i*_, so the calculation of the data set is shown in the following formula :

(1) $$\begin{array}{c} \text{set}=\sum_{l}\frac{t\cdot f}{n}x_{i}+A\cdot \frac{t\cdot f}{n}x_{i}{}^{2}+\xi . \end{array}$$

Among them, *A* is the creative fusion coefficient and *ξ* is the subjective coefficient of product design. ∑_*l*_*t* · *f*/*nx*_*i*_ represents the design collection of the cultural and creative products of sports events is the upgrade of sports event data; *t* · *f*/*nx*_*i*_^2^ represents the data collection of residents' health and an objective reflection of residents' fitness by the public.

In this study, the data set is 610, and the proportion of regional elements is 30%; the degree of creativity is 60%; and the guiding process in June,

**Assumption 2 .**

The survey time is *w*, the different groups is *g*, the age is *O*, the guidance degree is *C*, the regional index is *p*, and the design degree is *M*, then the calculation of the whole guidance process is shown in the following formula:

(2) $$\begin{array}{c} M=p\cdot \frac{\sum_{w=1,g=2}A\cdot g\cdot O}{C\left(1-p\right)}. \end{array}$$

Among them, *M*, *p*, and *g*, are classified indexes, *w* and *C* are continuous indexes; ∑_*w*=1,*g*=2_*A* · *g* · *O* represents the guidance of cultural and creative product design of sports events to residents' fitness; *C*(1 − *p*) represents the overall change of residents' fitness.

**Hypothesis 1 .**

The improvement effect of guiding situation is *H* that the difficulty of implementing guiding is tol: natural characteristics, historical characteristics, folk crafts, and regional culture are all greater than 30%, indicating that the design of cultural and creative products for sports events failed *c*_1_; natural characteristics, historical characteristics, folk crafts, and regional culture are all more than 60%, indicating that the design of cultural and creative products for sports events is normal *c*_2_; and natural characteristics, historical characteristics, folk crafts, and regional culture are all more than 80%, indicating that the design of cultural and creative products for sports events is successful *c*_3_. Therefore, the evaluation results of cultural and creative product design of specific sports events are shown in the following formula:

(3) $$\begin{array}{c} \text{tol}=a\cdot \frac{c_{1}}{\sum_{i=1}^{3}c_{i}}+b\cdot \frac{c_{2}}{\sum_{i=1}^{3}c_{i}}+c\cdot \frac{c_{2}}{\sum_{i=1}^{3}c_{i}}. \end{array}$$

Among them, *a*, *b*, and *c* are the adjustment coefficients of different evaluation degrees.

**Hypothesis 2 .**

Overall residents fitness assessment is *P*: natural characteristics is *P*_1_, regional culture is *P*_2_, historical characteristics is *P*_3_, folk crafts is *P*_4_, and complete the corresponding tests. Experts should compare before and after the test to find out the key points and factors of existing problems. The overall residents' fitness evaluation calculation is shown in the following formula:

(4) $$\begin{array}{c} p=\left(\frac{F_{1}+F_{2}}{\sum_{i=1}^{3}p_{i}}\right). \end{array}$$

With the help of provincial expert groups and authoritative organizations, from the perspectives of natural characteristics, historical characteristics, folk crafts, and regional culture, the cultural and creative products of sports events are designed, and the guiding investigation of residents' fitness is carried out. Then, an expert with more than 2 years' audit experience will be scored accordingly. At the same time, according to different residents, provide the corresponding cultural and creative product design of sports events, and finally, make a comprehensive evaluation.

The general group. According to the situation of regional residents, guide residents' fitness. At the same time, the fitness level of residents was investigated and comprehensively evaluated. According to the degree of residents' fitness guidance, this paper analyzes it properly, aiming at promoting the improvement of fitness levels.

SPSS21.0 software was used to analyze the data. Among them, the counting data is expressed by%, and the intergroup test is *X*^*2*^ test. $\bar{x}$ *±* *s* was used for measurement data, and *T* test was used for intergroup test. This paper analyzes the factors of residents' fitness promotion and finds out the improvement measures according to the analysis of influencing factors.

## 3. The Results and Analysis

### 3.1. Comparison of Natural Characteristics and Historical Characteristics

There is no significant difference between the two groups in implementing natural characteristics and historical characteristics after the design of cultural and creative products of sports events [19], the two groups are significantly better than before implementation, and there are significant differences. After the design of cultural and creative products of sports events, the natural and historical characteristics of the ordinary group are significantly better than those of the guiding group, and there are significant differences. The results are shown in Table 2.

The results in Table 2 are shown in Figure 3.

As can be seen from Figure 3, the amplitude of change between the ordinary group and the guide group is the same, but the amplitude of the guide group is slightly smaller than that of the ordinary group. Moreover, the mean value of the two groups is 5.5, which shows that there are differences between the two groups [20], and the results of the guiding group are better than those of the ordinary group.

The data in Figure 1 shows ups and downs, with the previous data lower than the average and the later data higher than the average, indicating that the comparison results of the two groups are constantly optimized and gradually due to the draw value. In addition, the variation of the numerical value is relatively uniform, and there is no significant change, which shows that the data analysis process is relatively stable. Therefore, the design of cultural and creative products of sports events of the guiding group meets the requirements, which can promote the improvement of residents' fitness level, especially natural culture, historical culture, folk crafts, and so on [21].

### 3.2. Comparison of Folk Crafts, Regional Culture, and Guidance and Prom Effects

After the design of cultural and creative products for sports events, the effects of regional culture and guidance promotion in the folk crafts of the ordinary group are better than those of the guidance group, and there are significant differences. The results are shown in Table 3.

The overall result is shown in Figure 4.

As can be seen from Figure 4, the overall judgment result is good. The local culture and folk craft of the two groups are better, and the numerical fitting degree and change range are better. Among them, the result of the numerical fitting degree is the best, followed by the change range. Although the numerical fitting degree is not good in the early stage, the fitting effect is good in the later stage. The range of numerical change also shows the characteristics of normal distribution, and the peak value is relatively low, which further illustrates the effect of guiding residents' health.

### 3.3. Influencing Factors of Residents' Fitness Guidance

The general clinical data of residents in the two groups and the indicators with significant differences in Tables 1 and 2 were assigned by single factor. The results are shown in Table 4.

The classification criteria in Table 4 are based on the critical values of different groups and relevant references [22]. At the same time, the data division standard adopts rounding and rounding to zero, and makes relevant comparisons [23]. Therefore, the results in Table 4 are relatively complete, mainly taking 60 points and 50 points as critical values.

### 3.4. Analysis of Influencing Factors Affecting Research Methods

Logistic Cox analysis is carried out with research methods as independent variables and indicators with significant differences as independent variables. The results are shown in Table 5.

It can be seen from Table 5 that natural characteristics, folk crafts, regional culture, and guiding promotion effect are all evaluation factors of residents' fitness guidance.

### 3.5. Safety Comparison of Cultural Creative Product Design in Sports Events

After observing the design of cultural and creative products of sports events for all middle-aged residents [24], it was found that 4 residents in the general group had decreased fitness effect, 2 had joint injuries and 1 had decreased physical function; one had accidental injury occurred in the guidance group. There was a significant difference in the incidence of complications between the two groups (*X*^*2*^ = 5.625, *P* = 0.018). After late rest, all the above-mentioned residents were relieved or recovered within 2∼3 days. The recovery effect of each resident is shown in Figure 5.

It can be seen from Figure 5 that although different patients exercise for residents, they will have different physical problems and injuries, which make them unable to exercise on time [25]. This study found that all residents will recover to varying degrees after a short rest. Moreover, the residents' physical recovery is basically the same, and there is no obvious difference. From the data in Figure 5, it can be seen that the impact levels of goals 1∼5 are all the same, and the levels are gradually increasing. This shows that the later development of residents' fitness is relatively stable. At the same time, the grade difference of different research objects is also consistent, that is, the grade difference is the same, which further shows that the guiding role of sports event culture innovation product design for residents' fitness is relatively stable. In addition, there is a linear correlation between residents' fitness levels and residents' research objects, which shows that the improvement of residents' fitness levels and the cultural innovation product design of sports events are positive. This shows that the design of cultural and creative products of sports events will improve residents' enthusiasm for fitness, but will not have a certain impact on their bodies. Therefore, the design of cultural and creative products in sports events will not only promote residents' fitness but also reduce residents' injuries in fitness.

### 3.6. Discussion of Research Results

Many factors, such as self-constitution, fitness awareness, and lack of effective guidance, will lead to unsatisfactory guidance of residents' fitness. The survey results show that the subhealth of Chinese residents is 12.4%, and the proportion is increasing year by year. The results show that residents' physical education has not been effectively implemented within 3∼4 months [26], and guidance will affect residents' graduation and improvement of physical fitness. The key to residents' fitness is to improve muscle function and shorten nerve reaction time. Lack of scientific implementation guidance will easily further affect the guidance of middle-aged residents, and their own random implementation methods will not have a good effect on guidance and promotion [22]. Therefore, looking for a scientific and effective implementation method is the key to improve the fitness guidance of residents, and it is also the focus of experts in the future.

The key to residents' fitness is to improve muscle function and shorten nerve reaction time. Lack of scientific implementation guidance will easily further affect the guidance of middle-aged residents, and their own random implementation methods will not have a good effect on guidance and promotion [27]. Therefore, looking for a scientific and effective implementation method is the key to improve the fitness guidance of residents, and it is also the focus of experts in the future. The key to residents' fitness is to improve muscle function and shorten nerve reaction time. Lack of scientific implementation guidance will easily further affect the guidance of middle-aged residents, and their own random implementation methods will not have a good effect on guidance and promotion. Therefore, looking for a scientific and effective implementation method is the key to improve the fitness guidance of residents, and it is also the focus of experts in the future. In addition, unsatisfactory residents' fitness guidance will affect the score of natural characteristics, folk crafts, historical characteristics, and guidance. In the post-implementation investigation, it was found that 4 residents in the general group had decreased fitness effect, 2 had joint injuries and 1 had decreased physical function, which further explained that the implementation of cultural and creative products designed for educational events would increase residents' fitness enthusiasm and arouse their interest in fitness, and had a light impact on their bodies. Some scholars' research shows that after the design of cultural and creative products for sports events, the scores of natural characteristics, historical characteristics and folk crafts of 45 residents have increased to 78.21 *±* 1.62 points, 20.19 *±* 1.14 points, and 20.63 *±* 1.92 points, which are significantly better than those of ordinary residents and consistent with the research results of this paper, further verifying the guiding and improving effect of cultural and creative products for sports events.

Among the residents in the two groups, there are significant differences in the indicators of single factor analysis, folk crafts, regional culture and guidance promotion effect, natural characteristics, and folk crafts are the evaluation factors affecting residents' fitness guidance. Among them, the OR of folk crafts and regional culture is 2.183 and 2.318, which may be poor with folk crafts, weak awareness of fitness among residents, and insufficient understanding of cultural innovative products. In addition, excessive exercise further aggravates muscle injury, reduces muscle and joint functions, and affects the design effect of cultural and creative products in sports events. In addition, when residents choose fitness methods in residents' fitness, they should first judge natural characteristics, folk crafts, and regional culture, so as to ensure the guiding and improving effect in the later period.

## 4. Conclusion

Cultural and creative product design of sports events is an additional industry of sports events, which can enhance the social influence of sports events, promote the development of residents' fitness and guide residents to actively engage in sports fitness activities. The design of cultural and creative products for sports events involves natural characteristics, folk crafts, regional culture, guiding and promoting effects, etc. It is necessary to deeply analyze the guiding effects of the above factors on residents' fitness. This article uses the regression analysis method to carry on the analysis, found that (1) the natural characteristic, the folk craft, the region culture, the guidance promotion effect are the main factor which affects the residents' fitness, will have the positive influence to the residents' fitness. (2) The regression analysis method has the high accuracy in the residents' fitness level analysis, the accuracy rate is above 90%, which is obviously superior to other algorithms. (3) The design of cultural and creative products in sports events should actively proceed from natural characteristics, folk crafts, regional culture, and guiding promotion effect, and formulate corresponding measures. However, there are still some deficiencies in this study, and there is no in-depth analysis of the relationship between design indicators and residents' fitness. In future research, we will focus on analyzing the internal factors of the cultural product design of sports events. The limitation of this study is that the amount of relevant data is relatively small, and the investigation time is short, which affects the accuracy and comprehensiveness of the research results. This study also has some deficiencies, mainly reflected in sports events cultural creative product design content, innovation level of research is insufficient, only research creative product design on the impact of residents' fitness, not different creative product design impact on the degree of analysis. Therefore, in future research, we will focus on the analysis of the above aspects.

## Figures and Tables

**Figure 1:** Relationship between supply and demand of cultural innovation product design in sports events.

**Figure 2:** Comparison of indicators of different groups.

**Figure 3:** Comparison of results of different groups.

**Figure 4:** Overall judgment result.

**Figure 5:** Late development of residents' fitness.

**Table 1:** General information of different groups.

Group	Content	Scope	Mean value
General group	Age	13∼56 year	Average age 43.21 ± 1.62 year
	Guidance situation	Effective guidance	16
		Invalid boot	4
	Degree of design	2∼6 Grade	Average design degree 4.22 ± 1.03
	Regional index	3.11∼3.45	Regional index 6.13 ± 1.0

Guide group	Age	12∼57 year	Average age 45.12 ± 2.33 year
	Guidance situation	Effective guidance	
		Invalid boot	15
	Guidance situation	Effective guidance	5
	Degree of design	2∼33 Grade	Average design degree 30.24 ± 1.07
	Regional index	3.01∼3.46	Regional index 6.25 ± 1.13

**Table 2:** The Comparison of natural and historical characteristics of residents in the two groups.

Group	Before implementation			After implementation		
	Natural characteristics (points)	Historical characteristics (points)	Folk arts and crafts (points)	Natural characteristics (points)	Historical characteristics (points)	Folk arts and crafts (points)
General group(*n* = 310)	56.33 *±* 5.21	62.61 *±* 6.42	78.34 *±* 5.27	82.71 *±* 6.22^ab^	56.49 *±* 11.24^ab^	50.13 *±* 9.82^ab^
Guide group(*n* = 310)	57.84 *±* 5.6	62.97 *±* 6.53	78.52 *±* 5.42	63.42 *±* 6.97^ab^	59.14 *±* 7.27^ab^	103.62 *±* 8.14^ab^
*T*	0.907	0.176	0.107	10.192	9.137	5.789
*P*	0.370	0.861	0.916	<0.001	<0.001	<0.001

Compared with that before implementation, ^*ab*^*P* < 0.05.

**Table 3:** Comparison of folk crafts, regional culture, and guiding promotion effect of residents in the two groups.

	Regional culture		Regional culture		Guide and improve the effect	
	General group	Modern folk crafts	Local culture	Foreign culture	Effective	Invalid
General group (*n* = 310)	198	182	176	174^ab^	178	222
General group (*n* = 310)	192	188	180^ab^	180	141^ab^	109^ab^
*T*	4.800		3.956		6.144	
*P*	0.029		0.047		0.013	

Compared with that before implementation, ^*ab*^*P* < 0.05.

**Table 4:** Indicators with significant differences.

Factors that differ	Threshold value
Natural characteristics (points)	<60 = 0, >60 = 1
Historical characteristics (points)	<60 = 0, >60 = 1
Folk arts and crafts (points)	<60 = 0, >60 = 1
Folk arts and crafts (points)	<50 = 0, >50 = 1
Guide and improve the effect	>50 = 0, <50 = 1

**Table 5:** Influence analysis of guiding influencing factors.

Correlation evaluation	*B*	Standard deviation	Wald	OR	*P*
Natural characteristics (points)	1.512	1.152	4.612	2.121(2.122∼2.492)	<0.01
Historical characteristics (points)	2.56	2.372	2.26	2.822(2.521∼2.933)	0.302
Folk arts and crafts (points)	2.473	2.238	3.929	2.183(2.102∼2.713)	<0.01
Regional culture	2.317	2.271	3.122	2.133(2.912∼2.26)	<0.01
Regional culture	2.426	2.447	2.627	2.823(2.482∼2.913)	<0.01

## Data Availability

The data used to support the ﬁndings of this study are available from the corresponding author upon request.
